# Bidirectional Neural Network Model for Glaucoma Progression Prediction

**DOI:** 10.3390/jpm13030390

**Published:** 2023-02-23

**Authors:** Hanan A. Hosni Mahmoud, Eatedal Alabdulkreem

**Affiliations:** Department of Computer Sciences, College of Computer and Information Sciences, Princess Nourah Bint Abdulrahman University, P.O. Box 84428, Riyadh 11671, Saudi Arabia

**Keywords:** visual field, bidirectional gated neural network model, glaucoma progression

## Abstract

Deep learning models are usually utilized to learn from spatial data, only a few studies are proposed to predict glaucoma time progression utilizing deep learning models. In this article, we present a bidirectional recurrent deep learning model (Bi-RM) to detect prospective progressive visual field diagnoses. A dataset of 5413 different eyes from 3321 samples is utilized as the learning phase dataset and 1272 eyes are used for testing. Five consecutive diagnoses are recorded from the dataset as input and the sixth progressive visual field diagnosis is matched with the prediction of the Bi-RM. The precision metrics of the Bi-RM are validated in association with the linear regression algorithm (LR) and term memory (TM) technique. The total prediction error of the Bi-RM is significantly less than those of LR and TM. In the class prediction, Bi-RM depicts the least prediction error in all three methods in most of the testing cases. In addition, Bi-RM is not impacted by the reliability keys and the glaucoma degree.

## 1. Introduction

Glaucoma is the leading cause of blindness worldwide and is characterized by irreversible retinal detachment (RTL) [1,2,3,4]. Embryonic stem cells and structural changes in the optic nerve head lead to progressive deterioration of the progressive visual field [2,3,4]. Assessment and classification of progressive visual fields is an important process for maintaining visual function. However, the progressive visual field test contains a lot of errors and random variations, so it may vary. This asymmetry in glaucoma is more severe than usual, making it difficult for doctors to understand the evolution of the progressive visual field [3,4,5,6]. The authors in [6], introduced rank-constrained spectral clustering with flexible embedding with a probabilistic neighborhood training phase process to compute the affinity matrix.

Research into machine learning algorithms used to assess glaucoma progression has attracted great interest and yielded impressive results. The authors [5] classified progressive visual field errors into 16 archetypes and determined their evolution. The author [6] reports an excellent classification using linear regression. However, only a few studies have attempted to analyze progressive visual field progression using deep learning algorithms. The authors [6] used a deep neural network to predict future progressive visual fields using a single progressive visual field test. The authors [7] used a variable auto-encoding (VAE) model to assess the progression of vision loss.

Convolutional neural networks are used for the sequential processing of time-dependent time series [8]. It has been used for sequence modeling for many years. RNNs can process current data using past data. RNN affects classification [9,10] according to the feature set, long-term memory (TM) [11], and gated repeated unit (GRU) [12] as two main target parameters in the RNN model long-term memory. It depends on the frame size. Our previous work showed that TM predicts future prospects better than traditional linear least squares regression [13]. In [14], the authors reported that magnetic theater arrays can capture local and global trends in the field of view over time.

Like MTs, GRUs can distribute activation blocks and interact with MTs more efficiently than conventional MTs [15,16,17]. Many studies in different fields have shown excellent results of GRU [18,19,20,21]. Recently, RNNs extended this method to include temporal learning and provide better context [20]. Because progressive visual field scans are also serial data with high internal correlation, bilateral unit repeats (Bi-MR) are better predictors of progressive visual field progression.

The contributions of this research are:

- This is the first study to use the Bi-RM model to detect progressive visual fields in glaucoma progression.
- The validation of the model performance in association with LR and TM models.
- The proposed Bi-RM depicted a higher predictive precision than LR and TM in all areas of progressive glaucoma prediction.
- Additionally, the Bi-RM model outperformed the other two models in the middle eye regions. These outcomes can be medically imperative to preserve the middle eye’s visual function.

## 2. Materials and Methods

This retrospective study was conducted on a public dataset of consecutive diagnostics at different times. The progressive visual field data used in this study were collected from the Glaucoma Database as depicted in Figure 1.

Dataset cases include at least 6 contiguous wild-type control cases with no duplicates in the database. In some cases, at least three years are needed between the 1st and 6th exams. For example, if there are 13 progressive visual field tests in a row, tests 1–6 are the first data, 7–12 tests are additional data. Test 13 was removed from the dataset. ^Tests^ 6 and 12 are for certification and the rest for training (Table 1). Table 1 contains information about the database.

### 2.1. Optometry of the Eye

Automated volume calculations were performed using the interactive threshold method (ITT) on a Humphrey Analyzer 950i (Medeie-tec, Inc., Dublin, CA, USA). Physiological cases of glaucoma are not included in the 54 (12-2) type test, but various other tests are used. The tone pattern gradually becomes 12-2. %FP < 41%, FN < 41% and loss of function <41% based on robust field testing.

### 2.2. Artificial Neural Network

We use two neural network models, TM and Bi-RM. Python version 3.8 (Google, Mountain View, CA, USA) with TensorFlow 2.3 is used to test predictions in this field.

#### Integrated TM Bi-RM

Single-layer neural networks are used to learn structural information from a given dataset with pre-processed input data. The definition of a neural network based on TM cells is as follows [2]:

(1) $$G1=G\left(z_{f}Y_{t}+z_{hf}h_{t-1}+a_{f}\right)$$

(2) $$G2=G\left(z_{i}Y_{t}+z_{hi}h_{t-1}+a_{i}\right)$$

(3) $$G3=G\left(z_{o}Y_{t}+z_{ho}h_{t-1}+a\right)$$

G1, G2, G3 are the gates.
$G\left(x\right)$ sigmoid formula.

where $z_{f},z_{i},\;z_{o},\;\mathrm{and}\;z_{C}$, $a_{f},\;a,\;a_{o},\;\mathrm{and}\;a_{C}$ The weights represent the bias parameters and the sigmoid is the activation function used in the network and can be written as

(4) $$G\left(x\right)=\frac{1}{1+e^{-Y}}$$

Inputs and outputs control the flow from the memory cell to the rest of the network by adding transition gates to the memory cell to shift the output of previous neurons to higher weights. Memory information is based on high activation frequency. When the signal from the input device is high, the information is stored in the memory cell. When the output unit is very active, it also sends information to another neuron. Otherwise, higher level information is stored in memory cells. The sigma body and the sun serve two different functional functions. where *h*(*t* − 1) represents the unit of the previous hidden layer and sums the weights of the three elements of the network. (4) Solving equation (C), _t_ is the unit current of the memory cell. Equation (5) shows the initial multiplication of the front cache block and the output of the front memory cell. The nonlinearity is added to the triple loading as a sigmoidal activation function, as shown in Equations (1)–(5). These are the previous and current steps of 𝑡 − 1.

GRU is a simple version of TM with only two ports, an update port and a reset port, which includes an access port and a forgotten port. The GRU has no additional memory cells to store information. That way, you only control the information on your device equations are adopted from our previous work in [2].

(5) $$U=G\left(z_{u}Y_{t}+z_{hu}h_{t-1}+a_{u}\right)$$

(6) $$R=G\left(z_{r}Y_{t}+z_{hr}h_{t-1}+a_{r}\right)$$

(7) $$\tilde{h_{t}}=tanh(zY_{t}+z\left(R⊗h_{t-1}\right)$$

An update port in Equation (7) defines the amount of updated information. In Equation (8), the relaxation gate corresponds to the update gate. If port is zero, read the input array and forget the previously computed state. It also performs $\tilde{h_{t}}$ the same function as a return module. $\tilde{h_{t}}\;$ℎ _❑ GRU la_ is a linear interpolation of the current and previous activation states from Equations (6) and (7) $h_{t-1}$

### 2.3. Process

The proposed method is a deep learning CNN, which consists of the following parts: an input layer, one convolutional layer used for sequence classification, and a dense layer. TM and Bi-RM neural networks are shown in Figure 2.

A single-layer time series neural network consists of six TM or RM binary cells connected in parallel. The first five cells receive 108 features as input, including 61 deviation values (DV), 61 sample values (PV), reliability data such as write loss rate and latency value. All inputs are normalized to an acceptable range to improve the performance of the deep learning model.

### 2.4. Purpose of the Activity

Square root value (mean square error) and absolute error as a measure of precision. It is calculated for each eye as Equations (8) and (9):

(8) $$SE=\sqrt{\sum_{i=1}^{n}\frac{{\left(Actual_{i}-predicted_{i}\right)}^{2}}{n}}$$

$SE\;\mathrm{is}\;\mathrm{mean}\;\mathrm{square}\;\mathrm{error}\;\mathrm{and}\;i=i^{th}\;\mathrm{test}\;\mathrm{point}\;\mathrm{of}\;\mathrm{visual}\;\mathrm{field}\;\mathrm{exam}$.

Absolute error (AE) for each test according to the formula:

(9) $$\begin{array}{c} AE_{n}=\sum_{i=1}^{m}\frac{\left|Actual_{i,z}-predicted{\;}_{i,z}\right|}{m}\\ z=z^{th}\;test\;point\;of\;visual\;field\;exam\\ i=i^{th}\;eye \end{array}$$

$predicted{\;}_{i,n}\;\mathrm{is}\;\mathrm{defined}\;\mathrm{as}\;\mathrm{the}\;\mathrm{total}\;\mathrm{deviation}\;\mathrm{value}\;\mathrm{of}\;i^{th}\;\mathrm{eye},\;z^{th}\;\mathrm{test}\;\mathrm{point}.$
*m* is the number of eyes.

Calculate the mean square error or *AE* for the *LR, TM,* and *Bi-RM* models using the formulas above. A one-way analysis of variance was performed to compare LR, TM, and Bi-RM. If the null hypothesis is rejected and the alternative hypothesis that the average difference is significant is accepted, a retrospective analysis is performed by matching and *p* < 0.05 is significant.

## 3. Results of the Experiment

Table 2 shows the demographic characteristics of the experimental database. The most common diagnosis is primary angle glaucoma (41.00%). The average classification time was 0.95 ± 0.84 years (Table 3). The average error measurement is shown in Table 3 and a typical sample of the absolute error progressive visual field test is shown in Figure 3.

Bi-RM classification results are better than LR and TM. Bi-RM has a mean square error of 3.71 ± 2.42 dB, while LR and TM are 4.81 ± 3.89 dB and 4.06 ± 2.61 dB, respectively. There is a significant difference in misclassification between the three models.

The eyes collected are shown in Figure 4. The Bi-RM misclassification margin for all eyes with greater than 50% coverage is 2 dB (530 eyes, 41.67%) and 2–3 dB (175 eyes, 13.76%). Corresponding LR ratings were 2 dB (329, 25.86%) and 2–3 dB (254, 19.97%), 2 dB TM (505, 39.70%), and 2–3 dB.

Out of 52 DV results, Bi-RM had the lowest misclassification of the three models. Bi-RM clearly outperforms LR and TM by 29 points (red dots) and 49 points (blue dots).

Table 4 shows the average classification error. The different parts of the field of view are shown in Figure 2 The progressive visual field is divided into six sections as described in [22]. The anatomy of the head of the optic nerve (regenerative, supranasal, temporal, nasal), the inferior temporal and inferior nasal (Figure 5), is shown in two parts (central and peripheral) (Figure 5). Bi-RM misclassification was significantly lower than LR and TM in all phases (*p* < 0.001).

The average values of mean square error classified by different factors are shown in Table 5 and Figure 6. Bi-RM classification error is significantly lower in false positives, false negatives, and fixed losses than the other two models. (*p* ≤ 0.025). Mean square error (average deviation) of the average deviation of the field of view can be seen. The classification error of the three models decreases as the average deviation value increases.

Classification errors and different sources are shown in Table 6 and Figure 7. (0.029) for all models (Figure 7).

## 4. Discussion

We proposed a Bi-RM model to detect and compute progressive visual fields. Validation of the accuracy of progressive visual field prediction using the Bi-RM network in association with LR and TM techniques. The Bi-RM model depicted the highest classification precision of the three models. The prediction mean error of LR, TM, and Bi-RM models are 5.71 ± 2.89 dB, 4.11 ± 2.71 dB, and 3.61 ± 2.32 dB. The mean error is considerably varied from the Bi-RM model and the other techniques (*p* < 0.002).

In all progressive visual field predictions, regions are partitioned into six parts according to the optic nerve composition, Bi-RM outperforms the other two techniques (*p* < 0.002). Bi-RM also depicts higher precision in the dominant and peripheral progressive glaucoma diagnosis (*p* < 0.002).

The classification performance depicts a deleterious correlation with false negative rate and fixation loss percentage in the compared methods; nevertheless, Bi-RM is the model least impacted by the deteriorating reliability metrics. As the average deviation lessened, the prediction precision will be reduced in the compared models, but the mean square error in Bi-RM is the least in the compared models. Bi-RM outperforms other models in advanced progressive glaucoma.

Many articles have employed deep learning to test the prediction of progressive glaucoma and its deviation. The authors in [23] constructed a deep-learning CNN to identify perimetric progression in glaucoma using a Softmax classifier. The area under the curve (AUC) is 92.6% for our proposed model, representing higher precision than machine learning networks. The authors in [24] predicted progressive glaucoma into 12 classes. In their continuation research, they investigated that the classes are correlated highly with the medical parameters of glaucoma. In [25], the authors focused on predicting the progressive angle of deviation rather than predicting eye arc deterioration.

The authors in [26] studied several machine learning models to identify glaucoma deviation utilizing the retinal nerve fibrous from tomography photography, the angle deviation, and the progressive eye examination.

In our research, we previously utilized the TM technique to predict and compute the progressive medical temporal exams including time sequences. In the current investigation, we employed a deep learning model using a Bi-RM model. Both GRU and TM are variants of the machine learning models, that utilize sequential input for temporal classification [27,28,29,30,31,32,33]. The authors in [16] proposed a GRU model to capture recurrent neurons to detect several temporal metrics. GRU and TM are alike as they include recurrent neurons in temporal modeling. Nevertheless, the GRU includes gated units that control the flow of input in the recurrent neurons excluding distinct memory [8,9,10,11,12]. The authors in [12] depicted that GRU is linked to the TM model in acoustic modeling. The authors in [18] proved that GRU has higher performance than TM with lower CPU time and higher error rate for audio recognition.

In our research, Bi-RM depicted a higher predictive precision than LR and TM in all areas of the progressive glaucoma prediction. In addition, the Bi-RM model outperformed the other two models in the middle eye regions. These outcomes can be medically imperative to preserve the middle eye visual function.

We also studied the CPU time for both training and classification time in comparison with the LR and TM models. Our model has half the training time as compared to the LR model and more than 60% less than the TM model. For the classification time, our model has the least time among the other models as depicted in Figure 8 and Figure 9.

## Figures and Tables

**Figure 1:** Example of a time shift sequence when 13 fields of view are implemented as in different eyes diseases [2].

**Figure 2:** Structure of the method proposed by TM. This model was previously published [13].

**Figure 3:** Typical example of average deviation (average deviation) progressive visual field classification in the first progressive visual field test. Five consecutive attempts to enter the field of view are shown from left to right, with the sixth attempt being the correct value.

**Figure 4:** Number of eyes ranked by root average square error (dB) (mean square error).

**Figure 5:** Field of view section. The six regions of the progressive visual field described by Garraway-Heath et al. [22] The progressive visual field is divided into central and peripheral areas. ST = total time; SN = supranasal. T = temporary. N = scarf, IT = fixed. IN = under the nose. *p* = endpoint. C = average value [2].

**Figure 6:** Mean classification error (mean square error) of different factors that are grouped together. (**a**) Mean square error versus false positive rate. (**b**) Mean square error versus false negative rates. (**c**) Mean square error versus capture loss ratio. (**d**) Mean square error and average deviation (average deviation) in the field of view. Bi-RM consistently showed the lowest false positive rate. Mean square error for LR, TM, and Bi-RM increased with decreasing average deviation. Other reliability indicators ignore linear relationships. LR = linear regression. TM = long-term memory. Bi-RM = bilateral repeat unit. Mean square error = root average square error.

**Figure 7:** Linear regression analysis between classification errors (mean square error) and different factors) Mean square error versus capture loss ratio in the field of view for Bi-RM = bilateral repeat unit..

**Figure 8:** Comparison of training CPU time.

**Figure 9:** Comparison of classification CPU time.

**Table 1:** Demographic features of the dataset.

Features	The Whole Dataset	Training Subset	Testing Subset
Count of cases	5595 (3593)	5313 (3311)	1161 (1161)
Average age	53.95	53.11	53.13
Standard deviation of age	±15.03	±15.99	±15.95
Mean first progressive visual field (dB)	−5.93 ± 5.11	−5.66 ± 5.15	−5.19 ± 5.33
Average progression years	5.53 ± 1.65	5.96 ± 1.96	3.51 ± 1.93
Average number of progressive visual field	6.36 ± 3.11	6.56 ± 3.33	5.99 ± 0.00
Mean deviation ≥−5.9 dB	3315	3596	919
−5 dB > Mean deviation ≥ −11 dB	1116	991	135
−11 dB > Mean deviation	1053	935	109
Data augmentation			
Total number of progressive diagnoses	9313	6051	1161
Average prediction time years	0.93 ± 0.63	0.91 ± 0.61	1.00 ± 0.93
Mean deviation ≥ −5 dB	5569	3651	919
−5 dB > Mean deviation ≥ −11 dB	1366	1131	135
−11 dB < Mean deviation	1156	1059	109

**Table 2:** Features of the dataset.

Cases	Count of Eyes
Males (%)	47.24%
**Outcome**	
Glaucoma	460
Starting acute deviation glaucoma	606
Pseudo deviation glaucoma	24
Initial deviation closure glaucoma	76
Subordinate glaucoma	90
Non-glaucoma	222

**Table 3:** Comparison of average mean square error and absolute error between LR, TM, and Bi-RM.

		LR	TM	Bi-RM	Analysis of Variance *p*-Value	Bonferroni Post Hoc *p*-Value		
						LR vs. Bi-RM	TM vs. Bi-RM	LR vs. TM
Classification error, average ± standard deviation	Mean square error (dB)	5.82 ± 2.89	5.06 ± 2.62	2.72 ± 2.42	<0.002	<0.002	<0.002	<0.002
	Absolute error (dB)	2.52 ± 0.56	2.20 ± 0.39	2.80 ± 0.36	<0.002	<0.002	<0.002	<0.002

Mean square error = root average square error; standard deviation = standard deviation; absolute error = pointwise average absolute error; LR = linear regression; TM = long short-term memory; Bi-RM = bidirectional gated recurrent unit.

**Table 4:** The classification error (mean square error) by progressive visual field sectors.

	Classification Error (Mean Square Error, dB), Average ± Standard Deviation			*p*-Value		
	LR	TM	Bi-RM	Bi-RM vs. TM	Bi-RM vs. LR	LR vs. TM
Superotemporal	5.83 ± 3.08	5.29 ± 2.86	5.02 ± 2.55	<0.002	<0.002	<0.002
Superonasal	3.55 ± 3.28	5.72 ± 2.76	5.32 ± 2.56	<0.002	<0.002	<0.002
Temporal	5.95 ± 3.52	5.79 ± 5.52	5.28 ± 2.92	<0.002	<0.002	0.220

**Table 5:** Mean classification error (mean square error) classified by reliability factor and average field of view deviation.

	Classification Error (Mean Square Error, dB), Mean ± Standard Deviation			Number of Eyes	*p*-Value			
	LR	TM	Bi-RM		Bi-RM vs. TM	Bi-RM vs. LR	LR vs. TM	Analysis of Variance
Classification error vs. false positive rate (false positive rate, %)								
False positive rate ≤ 2.5	5.90 ± 5.32	5.06 ± 2.65	3.72 ± 2.44	797	<0.002	<0.002	<0.002	<0.002
2.5 < False positive rate ≤ 5.0	5.74 ± 3.25	5.28 ± 2.69	3.80 ± 2.53	258	<0.002	<0.002	<0.002	<0.002
5.0 < False positive rate ≤ 7.5	5.32 ± 2.52	3.82 ± 2.38	3.52 ± 2.28	72	<0.002	<0.002	0.007	<0.002
7.5 < False positive rate ≤ 10.0	3.90 ± 2.28	3.73 ± 2.23	3.35 ± 2.94	57	<0.002	0.002	0.322	<0.002
False positive rate > 10	5.25 ± 3.29	5.29 ± 2.53	3.84 ± 2.33	88	<0.002	<0.002	<0.002	<0.002
Classification error vs. false negative rate (false negative ratio, %)								
False negative ratio ≤ 2.5	5.23 ± 3.88	3.58 ± 2.49	3.22 ± 2.22	766	<0.002	<0.002	<0.002	<0.002
2.5 < False negative ratio ≤ 5.0	5.26 ± 2.92	3.32 ± 2.79	3.20 ± 2.59	255	<0.002	<0.002	<0.002	<0.002
5.0 < False negative ratio ≤ 7.5	5.62 ± 3.02	5.05 ± 2.32	5.57 ± 2.06	209	<0.002	<0.002	0.007	<0.002
7.5 < False negative ratio ≤ 10.0	5.65 ± 2.92	5.52 ± 2.05	5.20 ± 2.89	92	<0.002	<0.002	<0.002	<0.002
False negative ratio > 10	8.32 ± 5.67	6.26 ± 3.03	5.94 ± 3.08	252	<0.002	<0.002	<0.002	<0.002
Classification error vs. fixation loss percentage (fixation loss percentage, %)								
Fixation loss percentage ≤ 2.5	5.92 ± 5.88	5.03 ± 2.74	3.66 ± 2.52	528	<0.002	<0.002	<0.002	<0.002
2.5 < Fixation loss percentage ≤ 5.0	6.54 ± 2.99	5.99 ± 2.20	5.27 ± 2.06	23	0.002	0.025	0.422	<0.002
5.0 < Fixation loss percentage ≤ 7.5	5.59 ± 2.87	5.08 ± 2.62	3.72 ± 2.38	275	<0.002	<0.002	0.002	<0.002
7.5 < Fixation loss percentage ≤ 10.0	3.95 ± 3.44	3.05 ± 2.29	2.86 ± 2.20	232	<0.002	<0.002	<0.002	<0.002
Fixation loss percentage > 10	5.98 ± 2.93	5.34 ± 2.50	3.98 ± 2.34	435	<0.002	<0.002	<0.002	<0.002
Classification error vs. average progressive visual field average deviation (average deviation, dB)								
Average deviation < −12	8.30 ± 5.56	6.98 ± 2.49	6.20 ± 2.69	230	<0.002	<0.002	0.273	<0.002
−12 ≤ Average deviation < −9	6.88 ± 2.86	6.57 ± 2.04	5.85 ± 2.20	80	<0.002	<0.002	0.229	<0.002
−9 ≤ Average deviation < −6	5.99 ± 2.44	5.43 ± 2.90	5.02 ± 2.80	242	<0.002	<0.002	0.002	<0.002
−6 ≤ Average deviation < −3	5.68 ± 3.97	3.70 ± 2.94	3.44 ± 2.72	278	<0.002	<0.002	<0.002	<0.002
−3 ≤ Average deviation	3.20 ± 3.22	2.28 ± 2.28	2.24 ± 2.27	542	<0.002	<0.002	<0.002	<0.002

**Table 6:** Statistical analyses indicating prediction error and reliability, and average angle of deviation using linear regression (LR).

	Correlation		LR			
	Spear Coefficient	Classification Error	Angle of Deviation	Diversion	$R^{3}$	Classification Error
Classification error vs. false positive rate						
LR	−1.036	0.566	−63	6.711	0.016	0.537
TM	−1.065	0.060	−61	6.186	0.003	0.068
Bi-RM	−1.063	0.156	−58	5.806	0.003	0.161
Classification error vs. false negative rate						
LR	1.666	<0.016	66.66	5.163	0.165	<0.016
TM	1.665	<0.016	56.67	3.603	0.356	<0.016
Bi-RM	1.668	<0.016	56.13	3.616	0.367	<0.016
Classification error vs. fixation loss percentage						
LR	1.085	0.005	11	6.636	< 0.016	0.636
TM	1.061	0.037	36	5.881	0.003	0.101
Bi-RM	1.066	0.006	37	5.676	0.006	0.053
Classification error vs. average progressive visual field Average deviation						
LR	−1.661	<0.016	−33.6	5.605	0.138	<0.016
TM	−1.665	<0.016	−36.5	3.656	0.583	<0.016
Bi-RM	−1.666	<0.016	−31.8	3.565	0.506	<0.016

LR = linear regression; TM = long short-term memory; Bi-RM = bidirectional gated recurrent unit.

## Data Availability

Data is available upon request.
